# Misfire Detection in Spark Ignition Engine Using Transfer Learning

**DOI:** 10.1155/2022/7606896

**Published:** 2022-07-08

**Authors:** S. Naveen Venkatesh, G. Chakrapani, S. Babudeva Senapti, K. Annamalai, M. Elangovan, V. Indira, V. Sugumaran, Vetri Selvi Mahamuni

**Affiliations:** ^1^School of Mechanical Engineering, VIT University Chennai Campus, Vandalur-Kelambakkam Road, Keelakottatiyur, Chennai-600127, India; ^2^Director CFC and CLT, SNS Group of Institutions, Coimbatore, India; ^3^Department of Mechanical Engineering, SNS College of Technology, Coimbatore, India; ^4^Department of Mathematics, Indira Gandhi College of Arts and Science, Kathirkamam, Puducherry, India; ^5^Department of Project Management, Mettu University, P.O.Box: 318, Metu, Ethiopia

## Abstract

Misfire detection in an internal combustion engine is an important activity. Any undetected misfire can lead to loss of fuel and power in the automobile. As the fuel cost is more, one cannot afford to waste money because of the misfire. Even if one is ready to spend more money on fuel, the power of the engine comes down; thereby, the vehicle performance falls drastically because of the misfire in IC engines. Hence, researchers paid a lot of attention to detect the misfire in IC engines and rectify it. Drawbacks of conventional diagnostic techniques include the requirement of high level of human intelligence and professional expertise in the field, which made the researchers look for intelligent and automatic diagnostic tools. There are many techniques suggested by researchers to detect the misfire in IC engines. This paper proposes the use of transfer learning technology to detect the misfire in the IC engine. First, the vibration signals were collected from the engine head and plots are made which will work as input to the deep learning algorithms. The deep learning algorithms have the capability to learn from the plots of vibration signals and classify the state of the misfire in the IC engines. In the present work, the pretrained networks such as AlexNet, VGG-16, GoogLeNet, and ResNet-50 are employed to identify the misfire state of the engine. In the pretrained networks, the effect of hyperparameters such as back size, solver, learning rate, and train-test split ratio was studied and the best performing network was suggested for misfire detection.

## 1. Introduction

In the modern era, transportation has become an integral part in the day-to-day life of every individual. People have to commute to places for either personal or official work. In one's income, transportation cost takes a reasonable amount of share. Also, from the industrial point of view, a huge amount of money is spent on transportation. While this is inevitable, there are few things that are in our hands by which one can save some amount of money. That can be done by keeping the vehicle in the proper working condition and thus saving the waste of money due to the faulty components and their working. Misfire is one such fault that takes away a lot of money and engine power. The causes for misfire may be due to any one of the reasons such as cylinder gasket leak, electrical fault, sensor malfunction, and defective spark plug. Misfire can result in loss of power and produce unwanted vibration that can impart wear and tear in allied components. Finding the misfire at an early stage and correcting it will save a lot of money for the owners of the vehicle. Misfire in an engine is not only a matter of money but also has the other technical impacts on the engine. In a multicylinder, if one cylinder is misfiring, then the remaining cylinders have to work extra in order to take the load of the engine. Apart from money and technical impact, misfire has an adverse effect on the environment also. Occurrence of misfire in a cylinder of the IC engine infers that the fuel has gone to the cylinder and the process of combustion did not initiate. Misfire can sometimes cause knocking, and the unburnt gases can be emitted as a pollutant into the atmosphere.

There are various misfire detection methods that are proposed by researchers and that can be categorized as follows [1]:

1. Temperature monitoring:
2. One can monitor the catalyst temperature [2] or exhaust temperature [3] and utilize these data for misfire detection; however, this method will work well only when the ignition-induced misfire rate is above certain percentage.
3. Wheel speed sensor:
4. Many researchers have worked on wheel speed sensor because the wheel speed sensor is already available in the automobile. Based on the patients in the crank speed, researchers find misfire in the engine [4].
5. Oxygen sensor:
6. It is mounted in the exhaust manifold, and from the fluctuation of the differentiated oxygen sensor signal, the misfire information can be found [5].
7. Pressure monitoring:
8. The misfire can be easily monitored effectively using the pressure inside the engine cylinder. However, the reliability and cost of the pressure sensor are the challenges [6–8].
9. Vibration monitoring:
10. Vibration signal acquired from the engine head is used for extracting features that can be used with machine learning algorithms. Babu Deva Senapati et al. have used how machine learning techniques along with features extracted from vibration signals and classified the misfire state of the IC engine [9]. There are researchers who have used the time domain in signals directly, and other researchers have transformed the time domain signals into frequency domain signals using fast Fourier transform, and then, they have applied machine learning for classification of the misfire states. However, vibration signals are highly dynamic in nature and complex. This throws a lot of challenges in the signal processing of vibrations.

Researchers have extensively used statistical features, histogram features, autoregressive moving average features, and wavelet features for misfire detection. While using these features, they have used a number of feature selection techniques including principal component analysis and decision tree. The classifiers they have used include decision tree support vector machine K Star algorithm and many more. While there are so many research works reported in the literature using machine learning in misfire detection, the effectiveness of machine learning depends upon the effectiveness of the features. The features engineering is very challenging especially when the signal is very complex like vibration signals. In this scenario, researchers look for some automated technology that can learn to classify without extracting explicit features from the signals. Deep learning is one such technology that has the capability to learn from the images without explicitly extracting features from them. However, one cannot take the pictures of the misfire inside the cylinder. It is unsafe and very costly affair.

Taking vibration signals from the engine cylinder head is a family and established activity. The vibration signals can be plotted and that can be used as a signature which can be used to detect the misfire in IC engines. Deep learning convolutional neural networks have a capability to understand the images and classify them as per the predefined classes. This study is our humble attempt to check whether the signatures of vibration signals plot are good enough to train deep learning algorithm for misfire detection. In the present study, pretrained networks such as AlexNet, VGG-16, GoogLeNet, and ResNet-50 were used. As these networks have been trained already for some other data set, they are called pretrained networks. It is easy to train pretrained network than a brand-new network from scratch. These pretrained networks have some knowledge, and we have to adapt that knowledge to the problem at hand (transfer the knowledge to other domain). This is called transfer learning, a subset of deep learning.

Later, significant developments in artificial intelligence (AI) and “Internet of Things (IoT)” have gained the attention of the scientific community. AI is considered as a powerful tool in the field of big data processing and data exploration. Modern intelligent fault diagnosis techniques are built on theories and concepts based on AI. Deep learning, an AI strategy first proposed by Hinton et al., in the field of science initiated the wave of research into different fields of study. Deep learning strategy (also termed as deep neural networks) consists of a number of neural layers stacked in a hierarchical structure that extracts information from the input. The architecture is called “deep” since the raw data information is learnt through multiple levels of layer-by-layer procedure. Starting from the raw data input, Deep Neural Network (DNN) discovers the structure of complicated data sets and automatically learns the most significant features through several layers. Automatic feature learning capability and improved nonlinear regression ability have made deep learning models to be widely used in language processing, object detection, visual inspections, surveillance, and robotics. Hence, there is a critical need and great potential to utilize the automatic learning capability of DNN in the field of mechanical systems fault diagnosis.

In the past few years, DNN was adopted by many researchers to either perform classification or feature selection in the field of fault diagnosis imitating traditional fault diagnosis methods. Initially, the features from acquired signals were extracted using various feature extraction techniques that are utilized to classify DNN models. Several authors reported on the above-mentioned strategy that is discussed as follows. A deep belief network was proposed by Li et al. to diagnose the condition of bearings and gearboxes using statistical features obtained from frequency, time, and time-frequency domains [10]. Chen et al. adopted a convolutional neural network (CNN) to detect the condition of the gearbox using frequency and time features [11]. An air compressor fault diagnosis was carried out by Verma et al. using a sparse autoencoder [12]. Shao et al. used an optimized deep belief network to diagnose bearing faults using 18 time features [13]. In this stage of fault diagnosis, DNN was used only as a replacement for the classifier, and the prime advantage of DNN feature learning was not equipped completely (Figure 1(a)).

After 2015, the researcher started using DNN for feature learning and feature selection along with classification. This provided a complete suite for all the activities in one go. Here, DNNs have taken images as input and corresponding classes as output. The DNNs are learnt without explicit need for feature extraction, feature selection, etc. The literatures based on the above-mentioned stage are discussed as follows. Condition monitoring of roller bearings was carried out by Guo et al. using deep convolutional neural networks consisting of two ensembles. Feature extraction and fault pattern recognition were carried out in one CNN while the fault classification was performed in the other CNN [14]. Zhao et al. performed tool condition monitoring using a convolutional long short-term memory (C-LSTM) [15]. Owing to the feature learning capability of DNN, the process of intelligent fault diagnosis grows into an effective and more automated approach (Figure 1(b)).

CNN forms the basic blocks of deep learning that have been adopted to learn complex features from image data. CNN is considered as one of the most dominant approaches in fault diagnosis, object detection, and speech recognition. However, very limited studies have been carried out in misfire detection of IC engines. Additionally, the application of CNN in the misfire detection was not attempted. Some related works representing the application of CNN in mechanical systems are presented in Table 1. In the present study, the performance of various state-of-the-art pretrained networks like AlexNet [23], VGG-16 [24], GoogLeNet [25], and ResNet-50 [26] was evaluated for detecting the misfire state from images acquired from vibration signals. Experiments were carried out on the pretrained networks by varying the train-test split ratio and various hyperparameters such as batch size, learning rate, and solver. The derived results are compared and tabulated to identify the suitable network for misfire detection in IC engine. The technical contributions in the present study are provided as follows.

- The present study considers four misfire conditions (c1 mis, c2 mis, c3 mis, and c4 mis) and one normal condition in a four-cylinder petrol engine.
- Vibration signals were obtained from the head of the engine, and the plots of vibration signals were utilized as input for pretrained networks.
- Four pretrained networks namely, AlexNet, VGG-16, GoogLeNet, and ResNet-50, were considered in the study to perform classification of misfire state.
- Various hyperparameters such as batch size, solver, learning rate, and train-test split ratio were altered, and the performance of the pretrained networks was assessed.
- The best performing network for misfire detection is identified based on the results obtained.

The rest of the paper is organized as follows. In Section 2, the experimental description includes experimental setup, data acquisition, and procedure.  Section 3 presents the overview of the convolution neural network (CNN).  Section 4 describes the process of transfer learning for misfire detection using vibration signal. Result and discussion are provided in Section 5, and the conclusion is presented at the end of the manuscript.

## 2. Experimental Studies

The present section discusses about the experimental setup fabricated for the study, data acquisition method, and experimental procedure followed in the study. The experimental setup comprises of a spark-assisted gasoline-powered IC engine. Initially, the accelerometer was placed (using adhesive technique) on the engine to acquire the vibration signals for good condition. The same procedure is repeated further to acquire the vibration signals of misfire in the IC engine by cutting off the spark in the cylinder one by one. The complete methodology involved in the process of misfire detection in IC Engine is depicted in Figure 2.

### 2.1. Experimental Setup

The present study utilizes a spark-ignited IC engine that has been equipped with provisions to create the misfire manually in a specific cylinder. The complete setup is connected to a data acquisition system and an accelerometer to acquire the vibration signals for every engine condition. An analog to digital converter helps in converting the acquired analog vibration signals into digital values that are stored in a storage device.  Figure 3 shows the experimental setup used in the present study. A 10hp-rated four-cylinder four-stroke spark-ignited (SI) engine is adopted in the present study. The misfire in the cylinders is performed by cutting off the power supply to the spark plugs present in each cylinder. A nut and screw mechanism is used to fix the accelerator in the engine at the specific position. The engine accelerator is firmly attached at the desired position via a screw and nut mechanism. The speed of the engine is kept constant in no-load condition. The specifications of the engine are provided in Table 2.

### 2.2. Data Acquisition

Data acquisition (DAQ) is the process of creating digital values from the world around such that it can be visualized, analyzed, and stored in a computer. In the present study, misfire detection in an IC engine is carried out by acquiring vibration signals with the help of an accelerometer (piezo-electric sensor with sensitivity of 10.26 mV/G). Accelerometers are capable of detecting both large and small vibrations. The working principle of the accelerometer states that output voltage magnitude is directly proportional to vibration signal intensity. The accelerometer is fixed on the centre of the engine block using adhesive techniques such that the vibration data are recorded for all conditions. A dactron FFT analyzer is used to convert the analog vibration signal into digital form. The acquired vibration data are further processed, and vibration plots are stored in a computer where a transfer learning approach is applied to identify the best performing pretrained network for misfire detection.

### 2.3. Experimental Procedure

Initially, electrical cranking was applied to start the engine at no-load condition. A buffer time of 15 minutes is provided to the engine for achieving the optimal operating condition. The FFT analyzer connected to the engine is turned on after engine stabilization. The engine speed was maintained at 1500 rpm, and the vibration data for normal operating condition are measured at 24 kHZ sampling frequency and 8192 sampling length. Five test conditions, namely, misfire in either of the cylinder 1, 2, 3, or 4 and normal condition, are considered in the study. Data acquisition for all the test conditions was performed at 1500 rpm.

The sample vibration signals for misfire and normal operating conditions are presented in Figure 4. The two waveforms acquired display significant differences aligning with the fact that unique patterns are displayed by vibration signals for each condition. The parameters considered during signal collection are described as follows:

- Sampling length: 8192 steps
- Sampling frequency: 24 kHz
- Number of instances for each condition: 100
- Speed: 1500 rpm

## 3. Description of Convolutional Neural Networks (CNN)

CNN formulates a connection between the image and image features by creating a set of biases and weights. The architecture is designed in a hierarchical manner that works on an automatic feature learning algorithm. The classification ability of CNN is based on the features that were learnt during the process of convolutions. The CNN architecture is composed of sequential stacking of several layers, namely, convolution layer, pooling layer, and fully connected layer. The general architecture of CNN architecture is provided in Figure 5.

The basic function of CNN is involved around the above-mentioned layer groups as given below:

- The input for a convolution layer is provided with the help of input layer which stores the image pixel values.
- The convolution layer is stacked next to the input layer that is filled with neurons of different weights and biases. The output of every neuron is calculated based on the product of volume and weights provided by the input. Rectified linear units (ReLU) is adopted widely as the activation function such that the nonlinearity among the problem is sustained.
- The immediate layer present next to convolution layer is the pooling layer which acts as the down-sampling layer. Features of high dimension are sampled down to achieve the spatial dimensionality such that the number of parameters can be reduced.
- The fully connected layers complete the CNN architecture by providing the classification results for a particular problem. The classification is carried out by assigning a particular range of values to every class such that improved performance is achieved. Matrix form of image features is converted into vector form through the fully connected layers.

CNN is able to transform the original input layer by layer to generate class scores for classification and regression purposes using convolutional and down sampling techniques. It is therefore important to remember that it will not be enough to simply determine the overall design of CNN architecture. These models can take some time to build and refine. Now, let us analyze the individual layers in detail, describing their hyperparameters and connectivity.

### 3.1. Convolution Layer

The learning process of CNN is instrumented by means of the convolution layer. The collection of several learnable kernels or filters is dependent on the parameters assigned to the layers. The kernels function in such a way that they spread across the wide range of input by consuming lower spatial dimensionality. In the process of convolution, two-dimensional activation maps are created for every image fed into the filter throughout the spatial dimensionality. The scalar product of weights and volume are calculated for every image data point that passes through the kernel present in the convolution layer. The values created through each filter (generally termed as activations) triggers the network to learn significant features that are available in the spatial domain. The midpoint of the kernel is placed over the input vector through which the weighted sum of itself and any neighboring pixels are calculated and replaced. Also, the model complexity can be reduced by convolution layers by means of hyperparameter optimization. Depth (no. of filters), stride (movement of filter in one direction), and zero-padding (adding zeros around the border of input image) are the three hyperparameters that can optimize the performance of convolution layers.

### 3.2. Pooling Layer

Pooling layers are equipped in deep learning architectures for the purpose of dimensionality reduction of particular data. Adoption of pooling layers can reduce the computational complexity of the model by shrinking the number of parameters involved. Pooling layer acts upon every value of input activation map and utilizes the “MAX” function for dimensionality scaling. Pooling layers have a destructive nature and are classified into two forms depending upon their function, namely, average and max pooling. Also, max pooling is the most widely used pooling layers due to the efficient performance on all data types. The size of the filter and stride length are commonly fixed at 2 × 2 to allow the pooling layer to expand throughout the input spatial dimensionality.

### 3.3. Fully Connected Layer

The ultimate layer of any CNN network is composed of fully connected layers. The output from the final convolution or pooling layer acts as the input to the fully connected layer. The output of convolution or pooling layers will be of matrix form which must be flattened before being fed into the fully connected layer. Sigmoid or softmax are adopted as the activation functions fully connected to perform the classification task for the given input data.

## 4. Misfire Detection in IC Engines Using Pretrained Models

The present section discusses about the various pretrained networks considered in the study to detect misfire in IC engines. Initially, the vibration signals are acquired for various conditions of IC engines and stored in the form of vibration plots (images). The acquired images are further resized and preprocessed to a size of 227 × 227 or 224 × 224 according to the input requirement of the adopted pretrained model. Further, various renowned pretrained network models like VGG-16, AlexNet, ResNet-50, and GoogLeNet were utilized to perform image classification and identify the condition of the IC engine. Transfer learning is adopted in this study in which the initial weights of the networks trained on ImageNet are restored. Also, to apply the networks for custom data set, the final output layers are replaced with new layers corresponding to the number of classes defined by the user.  Figure 6 represents the overall workflow of misfire detection in IC engines using pretrained networks. A brief description of the pretrained models considered in the study is provided as follows.

### 4.1. Data Set Formation and Preprocessing

In the present study, a data set of images containing the conditions of the IC engine was created from the vibration signals acquired. Five test conditions, namely, c1 mis, c2 mis, c3 mis, c4 mis, and normal condition, were considered. A total of 500 images (100 images for every class) were created using the acquired vibration signals. The acquired images were resized to a 224 × 224 or 227 × 227 such that the input size of the image is acceptable for the pretrained network adopted.  Figure 7 represents the vibration plots of various conditions of IC engine conditions collected for the study.

### 4.2. AlexNet Pretrained Network

Alex Krizhevesky introduced one of the best performing networks in the annual ImageNet Large Scale Visual Recognition Challenge (ILSVRC) that has been trained over 1.2 million images consisting of 1000 image classes. The network paved way for various advancements in the field of computer vision using deep learning. AlexNet is a simple network composed of 8 layers and 61 million learnable parameters. The input of the network accepts images of size 227 × 227. The input image is fed into the first convolution layer, where 96 different filters with a size of 11 × 11 try to convolve, normalize, and max pool the image to a size of 55 × 55. The output of the first convolution layer is fed into the second convolution layers consisting of 256 receptive filters followed by a max pooling layer of 3 × 3 size. The output image size is further reduced to a size of 27 × 27. The image is further reduced to a size of 13 × 13 while passing through the consecutive convolution layers (third, fourth, and fifth). Rectified linear units (ReLU) are adopted as the activation function in each layer to resolve nonlinear problems. Post the final convolution layer, two fully connected layers with 4096 learnable parameters is stacked to convert the image matrices into vector form. The architecture is completed with an output layer comprising of softmax activation function to perform classification for the adopted problem. To avoid the problem of model overfitting, a dropout layer of ratio 0.5 is added before the final fully connected layer.

### 4.3. VGG-16 Pretrained Network

The VGG-16 architecture was introduced by Karen Simonyan and Andrew Zisserman in the annual ILSVRC 2014 that was eventually claimed as the best performing network. The VGG-16 also termed as Visual Geometry Group-16 (also known as Oxford Net) was developed by a group of researchers from Oxford University. The network was constructed with 13 convolution layers, 5 max pooling layers, 3 fully connected layers, and a classification layer. The convolution layers are stacked in a unique pattern that is focused towards image classification problems. The working of the VGG-16 architecture can be understood by considering two learnable parameters “*B*” and “*d*” along with a filter of size 3 × 3. A mathematical operation is carried out when the image passes through the convolution layer which makes the filter to move about the image of “*z*” pixels such that the convolution operation is performed to produce an output image “*y*”. The following equation, *y*=*f*(*By*+*d*), represents the working of the convolution operation. Simple image features like edges are learnt by initial layers of VGG-16 architecture while complex image features are learnt by deep layers. The convolution process followed by max pooling helps in breaking down and resizing images such that highly contributing features are extracted along with limited memory consumption. The stride value and size of the filter can influence the image output from a convolution layer. Every convolution layer is provided with ReLU activation function, and a dropout of 0.5 is attached before the fully connected layer.

### 4.4. GoogLeNet Pretrained Network

In the annual ILSVRC 2014, Szegedy et al. proposed a network architecture named GoogLeNet that was aimed at solving image classification and object detection. The architecture was composed of 22 layers that had its application extended into the fields of facial recognition, robotics, adversarial training, etc. The network is arranged with nine inception modules connected to four convolution, four max pooling, three average pooling, five fully connected, and three softmax layers. ReLU is the activation function adopted in fully connected layers that are supported by a dropout layer of 0.5 ratio. Inception modules present in GoogLeNet architecture enable the network to solve more complex computer vision problems. Identification of complex features through variations in convolution layer filter size is the prime advantage of adopting inception modules. Such process can help in reducing the computational time and dimensional complexity. Even though the architecture of GoogLeNet looks robust with 22 layers, the volume of trainable parameters is less in comparison with AlexNet.

### 4.5. ResNet Pretrained Network

Residual network (ResNet) was the most successful and efficient network in the annual ILSVRC 2015 developed by He et al. The major advantages of using ResNet architecture is high convergence rate with accurate classification. The common objects in context (COCO) data set were used to train the ResNet architecture. Residual units were stacked together to form the ResNet architecture. ResNet architectures come in many forms depending on the number of residual units present and the variations in number of layers. ResNet architecture's success was influenced by the application of identity shortcuts in which the value of output identity mimics the input values identity. Like other networks, ResNet is also composed of convolution pooling and fully connected layers. The ResNet architecture resembles VGG network architecture. However, the former is eight times deeper than the latter resulting in a greater number of learnable features. Overall, the ResNet-50 architecture considered in the study consists of 49 convolution layers and 1 fully connected layer.  Table 3 represents the various characteristic features of the adopted pretrained networks.

## 5. Results and Discussion

In this section, the performance of the pretrained models (AlexNet, VGG-16, GoogLeNet, and ResNet-50) for misfire detection in IC Engine is evaluated. A total of four experiments were carried out based on variations in train-test split ratio, optimizer (or) solver, initial learning rate, and batch size. The overall experimentation was carried out in the desktop version of Matlab 2019b using the deep learning toolbox and transfer learning package. The detailed experimental study is explained as follows.

### 5.1. Effect of Train-Test Split Ratio

Train-test split ratio is the process of dividing the collected data set into two subsets, namely, training data and testing data. Training data are utilized to train our pretrained network while the testing data are used to evaluate the trained model for the custom data set. In the present study, five train-test split ratios were experimented for all the pre-trained networks by fixing default values for certain hyperparameters such that uniform evaluation is carried out. The hyperparameters like solver (SGDM), batch size (10), and learning rate (0.0001) were kept to default values to identify the best train-test split ratio.  Table 4 describes the performance of various pretrained networks for varying train-test split ratio.

From Table 4, one can infer that the performance of each pretrained network varies with a change in the train-test split ratio. The observations made from Table 4 state that AlexNet achieved a maximum accuracy of 90.70% for the train-test split ratios of 0.7. However, GoogLeNet and ResNet-50 achieve higher classification accuracy of 96.00% and 93.60% for train-test ratio of 0.75 and 0.8, respectively. Additionally, one can observe that VGG-16 pretrained network achieved 97.30% classification accuracy for 0.85 train-test split ratio. Computing the overall accuracy of the pretrained networks, it can be observed that VGG-16 produces the best classification accuracy of 95.76%.

### 5.2. Effect of Optimizers

Optimizers or solvers are the algorithms that are adopted during the training process such that the loss value is minimized to achieve an improved performance of the model. In the present study, an experimentation was carried out by varying the solvers, namely, stochastic gradient descent (SGDM), adaptive moment estimation (Adam), and root mean square propagation (RMSprop) to evaluate the performance of the model. The best performing train-test split ratio for each model was fixed based on the experimental results depicted in Section 5.1, i.e., 0.7 for AlexNet, 0.75 for GoogLeNet, 0.8 for ResNet-50, and 0.85 for VGG-16.  Table 5 depicts the performance of pretrained models for different solvers and load conditions.

Changing the optimizers can have an impact on the performance of the pretrained networks which is evident from Table 5. The observations state that the adoption of SGDM solver produced better classification accuracy for three pretrained networks, namely, AlexNet with 90.70%, VGG-16 with 97.30%, and GoogLeNet with 96.00%. However, ResNet-50 achieved a maximum accuracy of 97.20% for Adam optimizer. GoogLeNet displayed poor performance for RMSprop optimizer.

### 5.3. Effect of Learning Rate

Learning rate is one critical parameter that monitors the change in the training model with respect to the estimated error during every instance of model weight upgradation. Selecting the best learning rate can be challenging since small learning rate will elevate computational time while higher learning rates will result in improper training. In the present study, three values of learning weight like 0.001, 0.0001, and 0.0003 were used to evaluate the performance of the model. The other hyperparameters like train test ratio and optimizer are fixed for the pretrained networks that are depicted as follows: AlexNet (0.7 train-test split, SGDM solver), VGG-16 (0.85 train-test split, SGDM solver), GoogLeNet (0.8 train-test split, SGDM solver), and ResNet 50 (0.75 train-test split, Adam solver).  Table 6 depicts the performance of pretrained models for different learning rates.

From Table 6, one can infer that each pretrained network's performance varies with a change in learning rate. The observations state that AlexNet and VGG-16 achieved a maximum accuracy of 94.00% and 98.70% for 0.0003 learning rate, respectively. However, GoogLeNet and ResNet-50 achieved higher classification accuracy of 98.00% and 97.60% for learning rates 0.001 and 0.0001, respectively. Higher classification accuracy states that the model has learnt the features well and that the error value is minimal.

### 5.4. Effect of Batch Size

Batch size represents the number of samples that are propagated into a training network prior to model weight upgradation. The performance of the pretrained models in the present study is evaluated for different batch sizes (8, 10, 16, 24, and 32) with the selected best performing hyperparameters based on the experimental results mentioned in previous sections. The other hyperparameters like train test ratio, optimizer, and learning rate are fixed for the pretrained networks that are depicted as follows: AlexNet (0.7 train-test split, SGDM solver, and 0.0003 learning rate), VGG-16 (0.85 train-test split, SGDM solver, and 0.0003 learning rate), GoogLeNet (0.8 train-test split, SGDM solver, and 0.001 learning rate), and ResNet 50 (0.75 train-test split, Adam solver, and 0.0001 learning rate).  Table 7 depicts the performance of pretrained models for different batch sizes and load conditions.

From Table 7, one can observe that there are minimal changes incurred by changing the batch size. However, all the pretrained networks resulted better classification accuracy when the batch size selected was 10. Among all the networks, VGG-16 produced an overall accuracy of 98.08%. Increase in batch size will reduce the training time, thereby leading to accelerated training progress. However, the generalization capability of the network reduces with higher batch sizes. Thus, in the present study, batch size 10 is suggested as the optimal value for training the pretrained networks.

### 5.5. Comparative Study of Pretrained Models

In the present section, the performance evaluation of pretrained networks is discussed. Based on the experimental results obtained from previous sections, the optimal hyperparameters that enhance the performance of the pretrained models were identified. The list of best hyperparameters that produced an improved performance of pretrained models is provided in Table 8. The comparative study on the performance of pretrained networks with best hyperparameters is depicted in Table 9.

From Table 9, one can infer that VGG-16 established the utmost performance for the optimal hyperparameters selected. Based on the overall classification accuracy, superior classification, and lower computational time consumed, one can suggest VGG-16 for misfire detection in IC engines. The training progress and confusion matrix of best performing networks are presented in Figures 8 and 9, respectively.

From the training progresses represented in Figure 8, one can observe that the training process reaches saturation post 18 epochs. The sign of saturation represents that the VGG-16 network is trained effectively for the given IC engine misfire data set. The overall loss during the training progress for all the networks has drastically reduced representing the selection of optimal hyperparameters. Additionally, Figure 9 depicts the confusion matrix of VGG-16 architecture for misfire detection in IC engine. Confusion matrix in general depicts the performance level of a particular model or algorithm. The evaluation of the confusion matrix is carried out in regards to the instances classified in the major diagonal. The elements present in the major diagonal represent the correctly classified instances while the other nondiagonal elements depict the misclassified instances. The observations made from the confusion matrices state that VGG-16 architecture produced accurate classification accuracy for all conditions without any misclassifications except c4 mis (one instance is misclassified as c3 mis). Misclassification can occur due to various reasons like noise interruption, poor signal quality, and similarity between acquired signals. Lack of misclassification instances infers that the network has learnt all the features effectively and that the loss during training is negligible. Thus, from the observation made, VGG-16 is suggested as the best performing network for misfire detection in the IC engine. Additionally, VGG16 architecture consumed a computational training time of 2400 seconds in a low hardware system comprising of 8 GB RAM with no graphical card. However, the usage of sophisticated hardware systems (128 GB RAM with graphical card) can drastically reduce the computational time while elevating the capital cost of the system (up to 4 times).

### 5.6. Comparative Study with Other State-of-the-Art Works

A comparative study is carried out in this section to display the superiority of the proposed technique with other state-of-the-art works presented in the literature.  Table 10 displays the performance comparison of various techniques with the proposed technique. From Table 10, one can infer that the proposed method outclassed every other state-of-the-art works by displaying a classification accuracy of 98.7%. Classifier *k* nearest neighbor (KNN) exhibited the second-best classification accuracy with 95.8% next to that support vector machines (SVM), logistic model tree (LMT), and K-star algorithm with the value of 91.20, 89.40, and 82.60%, respectively.

## 6. Conclusion

In the present paper, four pretrained deep learning models, namely, AlexNet, VGG-16, GoogLeNet, and ResNet-50, were applied to diagnose the misfire in IC engine form vibration plots acquired. Four fault conditions (c1 mis, c2 mis, c3 mis, and c4 mis) and one normal condition were considered in the study. The pretrained networks are composed of CNN layers that perform an integrated approach of feature extraction, selection, and classification, thereby formulating an end-to-end machine learning approach. The pretrained networks are capable of processing the vibration plots and provide accurate classification results. The experimental results enumerate that the adopted networks are capable of learning complex features and produce convincing classification results for misfire detection in the IC engine. Various hyperparameters like train-test split ratio, optimizer, learning rate, and batch size were altered, and the optimal hyperparameters were identified for all the networks. VGG-16 was the best performing networks with 98.70% accuracy over AlexNet (94.00%), GoogLeNet (98.10%), and ResNet-50 (97.60%). Based on the comparative studies, VGG-16 is selected as the best performing network among the other networks considered in the study and is suggested for real-time application of misfire detection in IC engines. As a future scope, the position of the accelerometer and its effectiveness in classifying the cylinder correctly can be studied. Also, the proposed fault diagnosis system can be installed in real-time operation to perform on-board diagnosis.

## Figures and Tables

**Figure 1:** Stages of deep learning application in mechanical systems.

**Figure 2:** Overall methodology of fault diagnosis of misfire detection in IC engine.

**Figure 3:** IC engine experimental setup.

**Figure 4:** Sample vibration plots for (a) normal operation condition of IC engine and (b) misfire in cylinder 1.

**Figure 5:** General architecture of convolutional neural networks.

**Figure 6:** Overall workflow of misfire detection in IC engines using pretrained networks.

**Figure 7:** Vibration plots for normal condition in IC engine and misfire in cylinder 1, cylinder 2, cylinder 3, and cylinder 4.

**Figure 8:** Training progress of VGG-16 network for misfire detection in IC engine.

**Figure 9:** Confusion matrix of VGG-16 network for misfire detection in IC engine.

**Table 1:** Related works on deep learning-based methods for mechanical systems.

Reference	Deep learning technique	Mechanical system

[16]	CNN with wavelet transform	Motor bearing
[17]	Hierarchical CNN	Roller bearing
[18]	CNN	
[12]	Sparse autoencoder and deep belief network	
[19]	Recurrent neural network	
[20]	Stacked autoencoder	Gear box
[21]	Generative adversarial network	
[22]	CNN	Centrifugal pump

**Table 2:** IC engine specification.

Parameter	Specification

Manufacturer	Hindustan Motors
Fuel	Petrol (gasoline)
No. of cylinders	4
Alternator speed	1500 rpm
Power	7.35 kW
Bore diameter and stroke length	88.90 mm × 73.02 mm
Cooling system	Water cooled

**Table 3:** Characteristic features of adopted pretrained networks.

Model/network	Number of layers	Learnable parameters (in millions)	Input size of the image

AlexNet	8	60.0	227 × 227
VGG16	16	137.0	224 × 224
GoogLeNet	22	7.1	224 × 224
ResNet 50	50	25.7	224 × 224

**Table 4:** Performance of pretrained models for various train-test split ratios

Pretrained model	Classification accuracy for train-test split ratio (%)					Overall accuracy (%)
	0.60	0.70	0.75	0.80	0.85	

AlexNet	89.00	**90.70**	88.80	90.00	90.30	89.76
VGG-16	95.00	92.70	96.80	97.00	**97.30**	**95.76**
GoogLeNet	92.00	88.70	85.60	**96.00**	92.00	90.86
ResNet-50	84.00	86.70	**93.60**	89.00	84.00	87.46

The values highlighted in bold signify the best classification accuracy delivered by the pretrained model for the experimented train-test split ratio. While considering the last column, the best pretrained network with highest classification accuracy value is highlighted in bold.

**Table 5:** Performance of pretrained models for various solvers.

Pretrained model	Classification accuracy for different solvers (%)			Overall accuracy (%)
	SGDM	Adam	RMSprop	

AlexNet	**90.70**	88.70	80.00	87.29
VGG-16	**97.30**	90.70	92.00	**93.94**
GoogLeNet	**96.00**	95.00	69.00	87.71
ResNet-50	93.60	**97.20**	96.80	93.76

The values highlighted in bold signify the best classification accuracy delivered by the pretrained model for the experimented train-test split ratio. While considering the last column, the best pretrained network with highest classification accuracy value is highlighted in bold.

**Table 6:** Performance of pretrained models for various learning rates.

Pre-trained model	Classification accuracy for different learning rate (%)			Overall accuracy (%)
	0.0001	0.0003	0.001	

AlexNet	90.70	**94.00**	74.70	86.67
VGG-16	97.30	**98.70**	81.30	92.81
GoogLeNet	96.00	96.00	**98.00**	94.42
ResNet-50	**97.60**	96.00	94.40	**95.44**

Every pretrained network performs differently for the learning rates considered. The values highlighted in bold signify the best classification accuracies displayed by the pretrained networks for the variations in learning rate. The best performing network with highest overall classification accuracy is presented in the last column.

**Table 7:** Performance of pretrained models for various batch sizes.

Pre-trained model	Classification accuracy for different batch sizes (%)					Overall accuracy (%)
	8	10	16	24	32	

AlexNet	89.30	**94.00**	79.30	89.30	90.70	88.52
VGG-16	98.40	**98.70**	97.70	97.30	98.30	**98.08**
GoogLeNet	98.00	**98.10**	91.00	95.00	94.00	95.20
ResNet-50	96.00	**97.60**	83.20	93.60	97.40	93.56

Bolded values represent the best classification accuracy obtained by the individual pretrained networks for experimentation with different batch sizes. The pretrained network with best overall classification accuracy is represented in the final column.

**Table 8:** Optimal hyperparameters for pretrained model.

Pretrained model	Hyperparameters			
	Split ratio	Optimizer	Learning rate	Batch size

AlexNet	0.70	SGDM	0.0003	10
VGG-16	0.85	SGDM	0.0003	10
GoogLeNet	0.80	SGDM	0.001	10
ResNet-50	0.75	Adam	0.0001	10

**Table 9:** Performance comparison of pretrained models with optimal hyperparameters.

Pretrained networks	AlexNet	VGG-16	GoogLeNet	ResNet-50

Classification accuracy (%)	94.00	**98.70**	98.10	97.60

The values in bold signify the highest classification accuracy obtained by the pretrained network among all other networks considered post optimal hyperparameter tuning.

**Table 10:** Performance comparison with other state-of-the-art methods.

State-of-the-art methods	Classification accuracy (%)	References

KNN	95.80	[27]
Decision tree	80.60	[28]
LMT	89.40	[28]
SVM	91.20	[29]
K-star	82.60	[30]
Proposed method	**98.70**	

The proposed technique achieved higher classification accuracy (highlighted in bold) than other state of the art techniques presented in literature.

## Data Availability

The data used to support the findings of this study are included within the article and further data or information can be obtained from the corresponding author upon request.

## References

[1] Boguś P., Grzeszczyk R. (2001). Overview of engine misfire detection methods used in on board diagnostics. *J. KONES*.

[2] Tyree C. D. (1992). Emission levels and catalyst temperatures as a function of ignition-induced misfire. *SAE Technical Paper Series*.

[3] Tamura M., Saito H., Murata Y., Kokubu K., Morimoto S. (2011). Misfire detection on internal combustion engines using exhaust gas temperature with low sampling rate. *Applied Thermal Engineering*.

[4] Klenk M., Moser W., Mueller W., Wimmer W. (1993). Misfire detection by evaluating crankshaft speed - a means to comply with OBDII. *SAE Technical Paper Series*.

[5] Chung Y., Bae C., Choi S., Yoon K. (1999). Application of a wide range oxygen sensor for the misfire detection. *SAE Technical Paper Series*.

[6] Gu F., Jacob P. J., Ball A. D. (1999). Non-parametric models in the monitoring of engine performance and condition: Part 2: non-intrusive estimation of diesel engine cylinder pressure and its use in fault detection. *Proceedings of the Institution of Mechanical Engineers - Part D: Journal of Automobile Engineering*.

[7] Luján J. M., Bermúdez V., Guardiola C., Abbad A. (2010). A methodology for combustion detection in diesel engines through in-cylinder pressure derivative signal. *Mechanical Systems and Signal Processing*.

[8] Bahri B., Aziz A. A., Shahbakhti M., Muhamad Said M. F. (2013). Understanding and detecting misfire in an HCCI engine fuelled with ethanol. *Applied Energy*.

[9] Sharma A., Sugumaran V., Babu Devasenapati S. (2014). Misfire detection in an IC engine using vibration signal and decision tree algorithms. *Measurement*.

[10] Li C., Sánchez R. V., Zurita G., Cerrada M., Cabrera D. (2016). Fault diagnosis for rotating machinery using vibration measurement deep statistical feature learning. *Sensors*.

[11] Chen Z., Li C., Sánchez R. V. (2015). Multi-layer neural network with deep belief network for gearbox fault diagnosis. *J. Vibroengineering*.

[12] Verma N. K., Gupta V. K., Sharma M., Sevakula R. K. (2013). Intelligent condition based monitoring of rotating machines using sparse auto-encoders. *2013 IEEE Conference on Prognostics and Health Management (PHM)*.

[13] Shao H., Jiang H., Zhang X., Niu M. (2015). Rolling bearing fault diagnosis using an optimization deep belief network. *Measurement Science and Technology*.

[14] Guo X., Chen L., Shen C. (2016). Hierarchical adaptive deep convolution neural network and its application to bearing fault diagnosis. *Measurement*.

[15] Zhao R., Yan R., Wang J., Mao K. (2017). Learning to monitor machine health with convolutional Bi-directional LSTM networks. *Sensors*.

[16] He X., He Q. (2017). Energy-fluctuated multiscale feature learning with deep ConvNet for intelligent spindle bearing fault diagnosis. *IEEE Transactions on Instrumentation and Measurement*.

[17] Lee D., Siu V., Cruz R., Yetman C. (2016). Convolutional Neural Net and Bearing Fault Analysis. *Int’l Conf. Data Min*.

[18] Kang D. T., Kang H. J. (2019). Rolling element bearing fault diagnosis using convolutional neural network and vibration image. *Cognitive Systems Research*.

[19] Liu H., Zhou J., Zheng Y., Jiang W., Zhang Y. (2018). Fault diagnosis of rolling bearings with recurrent neural network-based autoencoders. *ISA Transactions*.

[20] Liu G., Bao H., Han B. (2018). A stacked autoencoder-based deep neural network for achieving gearbox fault diagnosis. *Mathematical Problems in Engineering*.

[21] Wang Z., Wang J., Wang Y. (2018). An intelligent diagnosis scheme based on generative adversarial learning deep neural networks and its application to planetary gearbox fault pattern recognition. *Neurocomputing*.

[22] Wen L., Li X., Gao L., Zhang Y. (2018). A new convolutional neural network-based data-driven fault diagnosis method. *IEEE Transactions on Industrial Electronics*.

[23] Krizhevsky B. A., Sutskever I., Hinton G. E. (2012). Cnn,” Commun. *ACM*.

[24] Simonyan K., Zisserman A. (2015). Very deep convolutional networks for large-scale image recognition. *3rd Int. Conf. Learn. Represent. ICLR 2015 - Conf. Track Proc.*.

[25] Asha P., Natrayan L., Geetha B. T. (2022). IoT enabled environmental toxicology for air pollution monitoring using AI techniques. *Environmental Research*.

[26] He K., Sun J. (2016). Deep Residual Learning for Image Recognition. https://arxiv.org/abs/1512.03385.

[27] Sumedh M., Devasenapati S. B. (2018). Misfire detection in I.C engines using machine learning approach” Pak. *Journal of Biotechnology*.

[28] Sugumaran A., Babu D. S. (2014). Misfire detection in an IC engine using vibration signal and decision tree algorithms. *Measurement*.

[29] Babu D. S., Noble G. A., Morganti C. R. (August 2010). Misfire detection in a spark ignition engine using support vector. *Machines”International Journal of Computer Applications*.

[30] Bahri A., Sugumaran V., Devasenapati S. B. (2013). Misfire detection in IC engines using K star algorithm. *International Journal of Research in Mechanical Engineering*.

